The article "Correlation between Selection of Time Window for Acute Cerebral Infarction and Efficacy of Intravascular Stent Implantation" was published in 2022. Journal: J Healthc Eng.

# Correlation between Selection of Time Window for Acute Cerebral Infarction and Efficacy of Intravascular Stent Implantation

**DOI:** 10.1155/2022/1357737

**Published:** 2022-02-08

**Authors:** Guanqing Feng, Yu Gong

**Affiliations:** ^1^Department of Neurology, the Ordos Central Hospital, Ordos City 017000, Inner Mongolia Province, China; ^2^Department of Interventional Medicine, Yantai Mountain Hospital, Yantai City 264003, Shandong Province, China

## Abstract

**Objective:**

To explore the correlation between selection of time window for acute cerebral infarction (ACI) and efficacy of intravascular stent implantation.

**Methods:**

The clinical data of 84 ACI patients treated in our hospital from March 2019 to March 2020 were selected for the retrospective analysis, all study subjects received intravascular stent implantation, and after discharge, patients were assessed by the Modified Rankin Scale (mRS) and divided into the good prognosis group (*n* = 46, mRS score ≤2 points) and poor prognosis group (*n* = 38, mRS score >2 points). The clinical data of patients in the two groups at admission underwent univariate analysis, the indicators presenting *P* < 0.05 were included in the logistic regression model, and the correlation between patients' treatment time window and clinical effect was analyzed by multivariate logistic regression analysis and linear fitting analysis.

**Results:**

According to the multivariate logistic regression analysis, low-density lipoprotein (LDL), time window, and blood glucose level before treatment were the independent factors affecting patients' treatment effect and were associated with the efficacy of intravascular stent implantation (*r* was 0.790, 0.889, and 0.672, respectively).

**Conclusion:**

LDL, time window, and blood glucose level before treatment are the important factors affecting the efficacy of intravascular stent implantation for ACI patients, among which the time window is most significantly associated with the clinical effect. Therefore, ACI patients should accept clinical treatment as early as possible.

## 1. Introduction 

Cerebrovascular diseases rank the first in the cause of death in China, among which acute cerebral infarction (ACI) accounts for approximately 80% [1]. Its pathogenesis is that various etiologies lead to occlusion of cerebral arteries, which induces ischemic and hypoxic necrosis of innervation. ACI is a disease with high morbidity, disability, and mortality, with a 19.04% incidence and 62.15% recurrence rate in China, ranking the top in the world. The world community has gradually recognized the severity of the disease and paid great attention [2]. At the onset of ACI, irreversible necrosis occurs in the ischemic core area, and the ischemic periphery is the ischemic penumbra with damaged neurological function but the neurons are still alive, so effective evacuation of the blocked blood vessels is the key to rescuing the ischemic penumbra [3, 4]. Intravascular stent implantation is considered as an alternative to traditional medical therapy for carotid dissection, which relieves luminal stenosis in the vessels by stenting, covers the torn portion of the arterial intima, prevents the formation of thrombus, and effectively stops the ischemic penumbra from developing into infarction or nerve cell necrosis [5, 6]. A clinical study pointed out [7] that atrial fibrillation, time window, and comorbid diabetes are important factors affecting the therapeutic effect of intravascular stent implantation, in which patients with comorbid diabetes will have intracranial vessel stenosis due to factors including abnormal blood composition, increased viscosity, and endocrine disorders, which affect treatment effect to some extent [8]. After the onset of cerebral ischemia, there is an allowed time when treatment can reduce the extent of brain damage, promote functional recovery, and improve long-term outcome, which is known as the time window. According to the Chinese Guidelines for Diagnosis and Treatment of Acute Ischemic Stroke 2018, the effective time window for rescuing the ischemic penumbra is within 4.5 h, and carrying out treatment within the time window can effectively evacuate the blocked blood vessels and restore blood flow, effectively avoiding irreversible brain tissue necrosis triggered by prolonged ischemia in ACI patients' brain cells [6, 9]. In this study, a clinically comparative study was conducted to explore the important factors affecting the efficacy of intravascular stent implantation and analyze the correlation between time window and patient outcome, so as to provide a reliable treatment basis for such patients.

## 2. Materials and Methods

### 2.1. General Data

A total of 84 patients treated in the Neurology Department of our hospital from March 2019 and March 2020 with an onset within 24 h were selected, and all of them had completed laboratory examinations including a biochemical test, routine blood test, and coagulation test before admission. The study met the World Medical Association Declaration of Helsinki (2013) [10].

### 2.2. Inclusion and Exclusion Criteria

Inclusion criteria: (1) all enrolled patients met the diagnosis criteria for ACI of the third revision in the second National Cerebrovascular Disease Academic Conference and were diagnosed with ACI after angiography, with clinical symptoms presenting as dizziness, hemiplegia, inarticulateness, vomiting, etc.; (2) patients were 18–75 years old; and (3) patients met the indicators of intravascular stent implantation (to be specific, (I) those without symptoms or had mild angina symptom, with the ECG and exercise stress test showing severe myocardial ischemia and coronary angiography indicating coronary artery stenosis >75%; (II) those with severe angina and unstable angina and coronary angiography indicating coronary artery stenosis >75%, which could not be alleviated with drug therapy; and (III) those who were confirmed to have vessel occlusion or severe stenosis and had blocked great vessels (carotid artery and/or middle cerebral artery).

Exclusion criteria: (1) patients had a history of cerebral infarction or suffered from stroke or myocardial infarction within 3 months; (2) patients had significant hemorrhagic diseases (such as drug allergic purpura, infectious purpura, thrombocytasthenia, and hemophilia) before or within the previous 6 months; (3) patients had a history of severe central nervous system damage (such as intracranial or spinal cord surgery and aneurysm); and (4) patients had bacterial endocarditis, acute pancreatitis, or severe kidney function obstacle.

### 2.3. Surgical Methods

All patients received the intravascular stent implantation. According to the treatment guideline for intravascular stent implantation [11] and with comprehensive consideration of patients' condition, the treatment was performed immediately after patients' family members had signed the informed consent. To ensure the homogeneity of the enrolled patients, treatment modalities such as stenting thrombectomy, arterial thrombolysis, and balloon dilatation were excluded, and intravascular stent implantation was adopted. Patients were lying flat on the operating table, after routine disinfection, draping, and local anesthesia, femoral artery puncture and sheathing were performed, 5F catheter was transmitted under wire guidance to the proximal end of stenosed artery for imaging, after determining the route, diameter, and length of stenosed lesion of the vessel, a suitable stent was selected and relieved precisely under wire guidance, after stent implementation, digital subtraction angiography (DSA) was performed to check the stent relief status and whether the remote vessel was smooth, and when the imaging showed that the stent was well placed, the catheter and wire were withdrawn, the arterial sheath was pulled out, and the puncture point was pressed [12]. Patients were repeatedly advised to lie on the back for 24 h, and 4 h after surgery, their activated partial thromboplastin time (APTT) was tested, and if it was within 50–70s, extubation could be performed, and then, the patients should lie on the back for another 24 h, with their puncture point being pressed for 6 h. Patients' various vital signs, including blood pressure, heart rate, breathing, and oxygen saturation were detected, and their urine volume was observed.

### 2.4. Assessment of the Prognostic Effect

The Modified Rankin Scale (mRS) [13] with the Spearman-related coefficient of 0.68 was adopted (see Table 1 for specific scoring criteria), with mRS score >2 points regarded as poor prognosis and mRS score ≤2 points regarded as good prognosis.

### 2.5. Statistical Methods

Statistical analysis was conducted by professional statistical software SPSS24.0, enumeration data were expressed by percentage (%), and measurement data were expressed by mean number ± standard deviation (Mean ± SD); for data consistent with normal distribution, the independent-sample *t*-test or analysis of variance was performed, and differences were considered statistically significant at *P* < 0.05; categorical variables were analyzed by the *X*^2^ test, and the level of statistical significance was defined as a two-sided test. Variables indicating *P* ≤ 0.05 and recognized effective variables in the univariate analysis entered the multivariate logistic regression model.

## 3. Results

### 3.1. Comparison of Clinical Data

Other than the mean age, treatment time window, hypertension, hyperlipidemia, low-density lipoprotein (LDL), and blood glucose before treatment, the clinical data between the two groups were not statistically different (*P* > 0.05), see Table 2.

### 3.2. Multivariate Logistic Regression Analysis

Taking whether patient prognosis was good or not as the dependent variable and including the single factors indicating *P* < 0.05 into the binary logistic regression model, the study results showed that LDL, blood glucose level before treatment, and time window were the independent factors affecting patient outcome, see Table 3.

### 3.3. Correlation between LDL and Clinical Prognosis

LDL was correlative with the mRS score (*r* = 0.790), see Figure 1.

### 3.4. Correlation between Time Window and Clinical Prognosis

Time window was correlative with the mRS score (*r* = 0.889), see Figure 2.

### 3.5. Correlation between Blood Glucose Value and Clinical Prognosis

For correlation between blood glucose value and mRS scores, see Figure 3.

## 4. Discussion

ACI refers to ischemic necrosis of brain tissue in its supply area caused by disturbance of cerebral blood circulation with high recurrence, high mortality, and high disability rates, which will leave patients with limb disability, language disability, and even dysphagia and dysuria, and some patients even experience cognitive dysfunction, seriously affecting the physical and mental health of patients. Interventional embolization is an effective treatment for ACI, and complex intracranial vascular obstruction requires stent assisted implantation [14, 15]. Free-radical-scavenging drugs given by intravenous infusion is the conventional regimen for the treatment of ACI. The drugs can improve the cerebral circulation and protect nerve cells, but will lead to increased or reduced platelet and elevated creatinine and then cause allergic reactions, so they should be used with caution in the elderly and those with liver dysfunction, restricting their clinical application to some extent. Intravascular stent implantation is a common method of interventional embolization, which improves ischemic symptoms in brain tissue by reducing the impact of blood flow on the vessel wall and increasing forward blood flow [16]. Because the stent placed has a certain stiffness and elasticity, it can partially change the route of the diseased artery, so that the vascular morphology and blood flow tends to be normal. Further clinical studies have confirmed [17] that stents can also promote the repair of the patients' vessel wall, and the stent mesh will be filled with new tissue to form a new lumen within the stent. The newly formed lumen is closer to the physiological lumen in terms of bending angle and diameter, which can increase the axial flow to some extent, so that the blood supply of the posterior circulation is improved [18]. In recent years, as the intravascular stent implantation technology is becoming more mature, it has been applied in treating diseases such as carotid artery, superior vena cava syndrome, and vertebrobasilar dolichoectasia [19] to benefit patients, gradually making it an important interventional treatment modality.

By analyzing the clinical data of patients in the poor prognosis group and good prognosis group, it was found that the mean age, treatment time window, hypertension, hyperlipidemia, LDL, and blood glucose level before treatment between the two groups were significantly different, and by including these factors into the binary logistic regression models, it was concluded that LDL, blood glucose level before treatment, and time window were the independent factors affecting patient prognosis. LDL transports neutral fat from plasma into peripheral tissue cells and can also be oxidized to form low-density lipoprotein cholesterol (LDL-C), which can induce the formation of foam in the blood followed by multiple arteriosclerotic biological effects, becoming an important factor predisposing to ACI [20]. In addition, the study found that patients' elevated blood glucose level before treatment was another important factor affecting clinical prognosis, which was consistent with the results of multiple studies [21]. Clinical studies have confirmed that increased blood glucose levels in the infarct area accelerate anaerobic glycolysis, leading to the production of a large number of acidic metabolites, which cause local paralysis and dilation of blood vessels and damage to the vascular endothelium. Elevated blood glucose level will increase the aggregation ability of red blood cells, reduce the blood flow rate, and promote platelet aggregation and adhesion, leading to the formation of thrombus [22]. The linear regression equation is the use of regression analysis in mathematical statistics to determine the interdependent quantitative relationship between two or more variables, where *r* is a statistical indicator first designed by Carl Pearson to indicate the amount of linear correlation between the studied variables, and *r* ≥ 0.8 is regarded as highly correlated [23]. The study results found that time window was highly correlative with the mRS score (*r* = 0.889). Clinical studies have found that there are two categories of outcomes faced by nerve cells corresponding to ACI, namely, cell necrosis and apoptosis, in which cell necrosis corresponds to neurons in a hypoxic state for up to 5 min, and apoptosis to ischemic penumbra cells, with lagging death time. According to the current findings, it is known that the pathological process of ACI includes loss of ionic balance, energy failure, activation of free radicals, and glial cell activation, so the later the intervention is initiated, the greater the degree of neurocellular pathophysiological alterations at the time of blood perfusion recovery [24]. The study findings showed that the time window was positively correlative with the mRS score, namely, the larger the time window, the higher the mRS score and the worse the clinical prognosis of patients. Therefore, timely treatment was the key to improving ACI outcome.

Study limitations: although the study included patients with ACI admitted to our hospital over a period of one year, the small sample size was still small and might have an impact on the findings; for the correlation study of the therapeutic effect, studies on infarct location, antioxidant drugs, and other factors can be added to explore the effect of other factors on the efficacy of intravascular stent implantation, and further refinement of the experimental design can benefit ACI patients more.

## Figures and Tables

**Figure 1:** Correlation between LDL and mRS score. The horizontal axis indicates LDL, and the vertical axis indicates the mRS score.

**Figure 2:** Correlation between time window and mRS score. The horizontal axis indicates time window, and the vertical axis indicates mRS score.

**Figure 3:** Correlation between blood glucose value and mRS scores. The horizontal axis indicates the blood glucose level value, and the vertical axis indicates the mRS score.

**Table 1:** Assessment standard of mRS.

Patients' condition	Scoring standard
No symptoms at all	0
No significant disability despite symptoms; able to carry out all usual duties and activities	1
Slight disability; unable to carry out all previous activities, but able to look after own affairs without assistance	2
Moderate disability; requiring some help, but able to walk without assistance	3
Moderately severe disability; unable to walk and attend to bodily needs without assistance	4
Severe disability; bedridden, incontinent, and requiring constant nursing care and attention	5

**Table 2:** Comparison of clinical data between the two groups.

Item	Good prognosis group (*n* = 46)	Poor prognosis group (*n* = 38)	*X* ^2^/*t*	*P*
Gender				
Male/female	24/22	20/18	0.002	0.967
BMI (kg/m^2^)	22.15 ± 1.20	21.71 ± 1.29	1.617	0.110
Mean age (mean ± SD, years)	54.07 ± 1.93	63.63 ± 3.08	17.341	<0.001
Treatment time window (mean ± SD, h)	3.33 ± 1.52	6.50 ± 1.75	8.884	<0.001
Drinking history	19 (41.30)	22 (57.89)	2.292	0.130
Smoking history	11 (23.91)	13 (34.21)	1.081	0.298
Combined underlying disease				
Hypertension	9 (19.57)	17 (44.74)	6.169	<0.05
Diabetes	8 (17.39)	7 (18.42)	0.015	0.902
Hyperlipidemia	3 (6.52)	10 (26.32)	6.233	<0.05
Total cholesterol (mean ± SD, mmol/L)	4.64 ± 0.27	4.70 ± 0.33	0.917	0.362
Uric acid (mean ± SD, *μ*mol/L)	291.63 ± 3.64	292.25 ± 2.81	0.859	0.393
Systolic blood pressure (mean ± SD, mmHg)	136.67 ± 7.04	136.66 ± 7.28	0.006	0.995
Diastolic blood pressure (mean ± SD, mmHg)	93.46 ± 5.43	93.29 ± 4.11	0.159	0.874
Triglyceride (mean ± SD, mmol/L)	1.04 ± 0.24	1.00 ± 0.21	0.804	0.424
LDL (mean ± SD, mmol/L)	3.47 ± 0.21	5.67 ± 0.24	44.796	<0.001
Blood glucose before treatment (mean ± SD, mmol/L)	4.42 ± 0.88	7.58 ± 1.05	15.009	<0.001
Educational degree				
College	4 (8.70)	2 (5.26)	0.370	0.543
Middle school	17 (36.96)	13 (34.21)	0.068	0.794
Primary school	25 (54.35)	23 (60.53)	0.324	0.569
Place of residence			1.248	0.264
Urban area	21 (45.65)	16 (42.11)		
Rural area	25 (54.35)	22 (57.89)		

**Table 3:** Multivariate logistic regression analysis.

Independent variable	OR value	95% CI	*P*
Time window	0.853	0.264–1.231	<0.001
Age	1.232	0.164–1.735	0.432
Hypertension	0.526	0.253–1.023	0.127
Blood glucose level before treatment	1.635	1.326–2.123	0.005
Hyperlipidemia	1.315	1.036–1.943	0.732
LDL	4.573	3.264–5.362	0.014

## Data Availability

Data supporting the findings of this study are available on reasonable request from the corresponding author.
